# Exploring Data Integrity of Dual-Channel Supply Chain Using Blockchain Technology

**DOI:** 10.1155/2022/3838282

**Published:** 2022-05-18

**Authors:** Wei Gan, Bo Huang

**Affiliations:** ^1^School of Business, Macau University of Science and Technology, Taipa 999078, Macau; ^2^School of Business, Guangdong Polytechnic of Science and Technology, Zhuhai 519040, China

## Abstract

The study intends to solve the problems of complex product circulation caused by information asymmetry and the untimely communication of production and sales information in the process of product sales to reduce the cost in the process of product circulation. Based on blockchain technology, the data integrity of the dual-channel supply chain is studied. First, the data of the supply chain conduct coordinated management to achieve the integrity of the supply chain data. Then, under the background that both retailers and suppliers are risk-neutral individuals, the benchmark model of the dual-channel supply chain is constructed, and the online and offline sales prices of products under different decision-making modes are analyzed. Finally, taking fresh agricultural products as an example, the sales strategies of the online and offline sales channels of fresh agricultural products are studied, and a dual-channel supply chain model is constructed. The profit of each member in the supply chain system under this model is obtained by the inverse method. The simulation results demonstrate that the retailer's revenue and the total revenue of the system increase obviously with the growth of the price discount coefficient after the price discount strategy is applied. When the compensation cost is between 1,000 and 3,000, the profit of retailers in the supply chain system is improved by using the price coordination mechanism, while the profit of suppliers decreases to some extent. When the value of compensation cost is 7,000–9,000, the application of the price coordination mechanism increases the profit of suppliers in the supply chain system, while the profit of retailers declines to a certain extent. The research content reported here effectively alleviates the profit conflict and the double marginal effect between the two channels and enriches the theoretical system knowledge of the coordination of the two channels' supply chain of agricultural products.

## 1. Introduction

Under the background of the rapid development of a free-market economy, to realize the modernization of China's agricultural field, it is essential to keep up with the pace of reform and opening up. In terms of emerging technologies, the development of the Internet has brought enormous convenience to the production and circulation of agricultural products and other links [1]. However, under the influence of the traditional domestic sales model, the main circulation model of agricultural products of China is still offline sales. This type of sales is dominated by intermediary businesses and wholesale markets and has certain limitations in terms of efficiency and brand appeal. However, the online sales platform makes up for these disadvantages and has brought greater development space for brand publicity and standardization innovation of agricultural products [2, 3]. The online sales platform not only saves consumers' time and enriches consumers' purchase channels but also solves the problems caused by information asymmetries, such as the imbalance of production and marketing in the sales process of agricultural products and excessive links in the circulation process. Therefore, the dual-channel supply chain model is the main trend of the development of the supply chain of agricultural products in the future [4].

The dual-channel supply chain model combines online transaction channels based on Internet platforms and offline circulation channels based on entity enterprise. In terms of the traditional dual-channel supply chain coordination, Qi et al. [5] described the coordination problem of the dual-channel supply chain as a supplier's Stackelberg game model, which obtained optimal pricing decisions and corresponding profits in centralized and decentralized systems. To improve the performance of the decentralized system, the authors proposed an online channel price discount contract and an offline channel price discount contract to coordinate the two-channel supply chain. Meanwhile, they provided a transfer payment mechanism to realize the win-win situation of both sides. Zhang et al. [6] considered a dual-channel supply chain system composed of a single manufacturer and a single retailer to study the influence of advertising cooperation on dual-channel supply chain decision-making. They also analyzed the advertising investment level and supply chain profit of centralized and decentralized dual-channel supply chains based on the Stackelberg game model. Then, they constructed the decision-making model of dual-channel supply chains under different contracts to analyze how manufacturers optimized profits of both sides through an effective coordination mechanism. The emergence of technologies such as cloud computing, big data, the Internet of Things (IoT), and blockchain has accelerated the development of society towards automation and intelligence. Miraz and Ali [7] pointed out that blockchain technology was a distributed ledger technology composed of various data combinations. Simply speaking, it is jointly maintained by all participants. The unique construction model and new information technology build a strong asset trust relationship and value transmission network, which makes the blockchain have the functions of being distributed and tamperproof, and value can be transmitted. Chen et al. [8] proposed that in this low-trust market competition environment, blockchain had built a good trust management mechanism with its special new model, which had quietly changed the operating environment of the financial industry.

Dual-channel supply chains have brought great benefits to consumers and reduced the loss in the process of commodity circulation, but the opening of online transaction channels will inevitably bring some impact on the traditional sales model. Based on blockchain technology, the data integrity of the dual-channel supply chain is studied. First, the data of the supply chain conduct coordinated management. Second, under the background that both retailers and suppliers are risk-neutral individuals, the benchmark model of the dual-channel supply chain is constructed, and the online and offline sales prices of products are analyzed under different decision-making modes. Finally, taking fresh agricultural products as an example, the sales strategies of the online and offline sales channels of fresh agricultural products are studied, and a dual-channel supply chain model is constructed. The innovation of the research lies in the introduction of revenue sharing and price discount contract strategies to implement coordinated management of the supply chain. It can promote the supply chain system revenue to reach the optimal state as much as possible and obtain the corresponding price equilibrium solution and contract parameters. Moreover, it is verified that such contract parameters that can improve the efficiency of the supply chain must exist.

## 2. Construction of the Dual-Channel Supply Chain Model Based on Blockchain Technology

### 2.1. Blockchain Technology

#### 2.1.1. Infrastructure

Blockchain is composed of six layers, including the data layer, network layer, consensus layer, incentive layer, contract layer, and application layer. These six layers are combined from top to bottom to realize the concretization of function allocation. The six layers cooperate with each other to ensure the smooth and safe operation of the whole blockchain [9, 10]. Among them, the data layer, network layer, and consensus layer are the three indispensable layers in a standardized blockchain network, while the other three layers can be designed according to specific practical needs.  Figure 1 displays the blockchain infrastructure.

In Figure 1, the bottom layer is the data layer primarily describing the physical characteristics of the blockchain network, which is the most critical data structure in the whole blockchain architecture. The main feature of the data layer is that data can be fully backed up and data information cannot be tampered with [7]. This layer structure records information such as timestamp, address, and public and private keys, as shown in Figure 2.

The network layer is principally responsible for the information exchange in the whole blockchain to realize the information receiving and sharing among nodes in the blockchain network. Each node in the blockchain network can not only receive information but also proinformation. After creating a new block, each node will inform other nodes in the network structure through broadcast, and the new block created needs to receive verification from other nodes. When the pass rate after verification is higher than 51%, the new blocks created can be added to the backbone structure [11, 12].

Based on the availability of blockchain data, the consensus layer enables highly dispersed nodes in a decentralized system to reach consensus. As one of the core technologies in the blockchain structure, consensus mechanisms can have a certain impact on the security and reliability of the entire blockchain structure. Moreover, these consensus mechanism algorithms are encapsulated in the consensus layer structure [13]. By providing a certain reward distribution mechanism, the incentive layer motivates each node in the blockchain to mine and participate in the verification of new blocks. The smart contract layer is the programmable and trustless foundation in the blockchain. It specifies the transaction methods and processes in detail, including various scripts and codes, and has the characteristics of automatic execution and tamperproof. The application layer is responsible for docking with various application scenarios, covering all entities in the application scenarios, and completing the entire business logic according to the rules formulated by smart contracts.

#### 2.1.2. Consensus Mechanism

The consensus mechanism can be regarded as a vote between each node in the blockchain. Each node in the blockchain verifies and approves the recently generated transaction information through the specific consensus mechanism, and on this basis, the service delay can be minimized. If transaction data lead to consensus among several nodes in the entire blockchain structure, it can be considered that the data can also lead to consensus across the entire network. Proof of Work (PoW) and Proof of Stake (PoS) are the mainstream consensus algorithms.

In the PoW mechanism, each node solves the complex Secure Hash Algorithm 256 (SHA256) problem according to its computation force, as shown in the following equation:

(1) $$\begin{array}{c} H\left(n\left\|\;\right.h\right)\leq t. \end{array}$$

In equation (1), *H* denotes the Hash function, *n* stands for a random number, and *t* represents the target difficulty. As can be seen from equation (1), the smaller the target difficulty value, the fewer random numbers that meet the conditions. Each node in the blockchain competes with each other to find random numbers that meet the conditions, and the node that spends the least time in the search process gets the right to account [14].

The PoW mechanism has disadvantages such as low efficiency and high energy consumption. Given this deficiency, relevant scholars put forward the PoS mechanism. In this mechanism, there is no need for complicated calculation, thus saving a wealth of power resources. The basic principle of the PoS mechanism is to select the node with the largest ownership proportion among all network nodes participating in the competition for the corresponding operation. This mechanism believes that the shares of nodes have a certain impact on the difficulty of generating the latest block, as shown in the following equation:

(2) $$\begin{array}{c} H\left(n\left\|\;\right.h\right)\leq s\left(M\right).t. \end{array}$$

In equation (2), *s*() refers to the equity return function. According to equation (2), when the target difficulty is maintained at a certain value, the share of absenteeism will have a certain impact on the calculation difficulty of random numbers.

#### 2.1.3. Smart Contracts

The idea of smart contracts emerged almost at the same time as the Internet. The term “smart contracts” was first proposed by the famous American scientist Nick Szabo. Its essence is similar to conditional statements in programming. To be specific, the developer needs to set a precondition in advance. When the precondition is satisfied, the smart contract will be triggered and the instructions in the smart contract will be executed to realize the “intellectualization” of the contract. Smart contracts have gained extensive attention and development only after the emergence of blockchain technology. In a blockchain system, smart contracts can cooperate with a consensus mechanism to build a decentralized system and prevent data from being tampered with at will. Smart contracts have now become an essential feature of blockchain technology.

From the perspective of programming, the smart contract in a blockchain system is essentially a piece of instruction code. However, compared with the conventional instruction code, it has many constraints. For example, smart contracts have difficulty accessing off-chain data such as weather information and competition results; they cannot exceed resource limits; they also consume large amounts of resources when executing code. Due to the above constraints, smart contracts can only control transaction resources on the ecological chain at present.

Because of its unique nature, blockchain can be applied to the Internet of Things, financial statistics, donation tracking, inventory tracking, data storage, healthcare, and many other fields. Applications of blockchain in each domain have their specific business processes, which require service providers to build new custom blockchains to meet the particular service requirements. In today's environment of explosive data growth, the main challenges faced by blockchain are the expansion of the scale of the blockchain network and the number of users it can support. Besides, it is essential to reduce the delay because the implementation of functions in blockchain-based applications depends on consensus. In addition, the response time needs to be reduced, which fundamentally relies on the improvement of the consensus algorithm. Moreover, it is necessary to ensure network security by using devices that have limited resources and cannot perform heavy tasks to protect the network and effectively prevent malicious nodes from damaging the network.

### 2.2. Two-Channel Supply Chain Benchmark Model

#### 2.2.1. Problem Description

Assuming that the market demand is uncertain, a dual-channel supply chain composed of a retailer and a supplier is considered here. In this structure, the supplier occupies the main position. Therefore, the supplier can give priority to determining the green degree and wholesale price of a product according to its demand, and the retailer determines the offline retail price according to the wholesale price determined by the supplier [15–17]. In addition, in the dual-channel supply chain, suppliers can sell their products through online and offline channels, as shown in Figure 3.

#### 2.2.2. Model Hypothesis and Parameter Description

Webb proved in 1994 that products have a certain impact on the natural environment, pointing out that products are produced in accordance with certain natural guidelines, recycling certain components where possible. The concept of a green supply chain was first proposed in 1996, and it appeared in an “Environmentally Responsible Manufacturing (ERM)” conducted by the Manufacturing Research Association of Michigan State University. Its main content is to take environmental impact and resource efficiency into consideration during the operation of the entire supply chain and ultimately achieve the goals of minimum environmental impact and highest resource utilization efficiency. With the intensification of environmental problems, the research on the green supply chain has received extensive attention from all walks of life. Meanwhile, the research on the green supply chain in academia has become more and more in depth, and surprising results have been achieved.

Hypothesis 1: in the case of uncertain market demand, it is assumed that the improvement of product greenness can effectively increase market demand, and consumers of online and offline sales channels have the same preference for green products [18]. Demand functions of online and offline sales channels can be expressed as follows:
  (3) $$\begin{array}{c} D_{e}=s\left(a+\varepsilon \right)-p_{e}+\theta p_{r}+\eta \tau ,\\ D_{r}=\left(1-s\right)\left(a+\varepsilon \right)-p_{r}+\theta p_{e}+\eta \tau , \end{array}$$
where *D*_*e*_ represents the product demand of online sales channels, *D*_*r*_ refers to the product demand of offline sales channels, *a* signifies a constant and *a* > 0. Besides, *ε* represents the random demand caused by market uncertainty and *ε* ~ *N*(0, *σ*^2^); *s* denotes retailers' share of the offline market and 0 < *s* < 1; *θ* signifies the coefficient of cross elasticity of online and offline sales channels; *p*_*e*_ stands for the online sales price of the product; *p*_*r*_ indicates the offline sales price of the product; *η* represents consumers' preference coefficient for green products and *η* > 0; *τ* refers to the green degree of products and *τ* > 0.
Hypothesis 2: assume that the cost of product greenness borne by the supplier is 1/2*ρτ*^2^, where *ρ* represents the green cost coefficient per unit.
Hypothesis 3: assume that the cost of production per unit of product is *c*, the wholesale price determined by the supplier is *w*, and the costs of both the supplier and the retailer are 0. Besides, *p*_*r*_ > *w* > *c* > 0 and *p*_*e*_ > *w* > 0.
Hypothesis 4: suppliers will try their best to avoid shortages, so there is no upper limit on production capacity, and there is no difference in product quality between online and offline sales channels [19, 20].
Hypothesis 5: there is no information asymmetry in the supply chain structure, information is shared, and retailers and suppliers are risk-neutral individuals. Moreover, the profit is denoted as Π_*j*_ and the expected profit as *E*Π_*j*_. Besides, the expected utility is represented by *E*Π_*j*_, where *j* ∈ {*z*, *g*, *r*}, among which *z* represents the whole supply chain, *g* represents the supplier, and *r* refers to the retailer.

Based on the above assumptions, the profit function of suppliers and retailers can be defined as follows:

(4) $$\begin{array}{c} \Pi_{g}=\left(w-c\right)\left[s\left(a+\varepsilon \right)-p_{r}+\theta p_{e}+\eta \tau \right]+\left(p_{e}-c\right)\left[\left(1-s\right)\left(a+\varepsilon \right)-p_{e}+\theta p_{r}+\eta \tau \right]-\frac{1}{2}\rho \tau^{2},\\ \Pi_{r}=\left(p_{r}-w\right)\left[s\left(a+\varepsilon \right)-p_{r}+\theta p_{e}+\eta \tau \right]. \end{array}$$

The expected profit of suppliers can be written as follows:

(5) $$\begin{array}{c} E\left(\Pi_{s}\right)=\left(w-c\right)\left(sa-p_{r}+\theta p_{e}+\eta \tau \right)+\left(p_{e}-c\right)\left[\left(1-s\right)a-p_{e}+\theta p_{r}+\eta \tau \right]-\frac{1}{2}\rho \tau^{2}. \end{array}$$

Equation (6) describes the expected profit of retailers:

(6) $$\begin{array}{c} E\left(\Pi_{r}\right)=\left(p_{r}-w\right)\left(sa-p_{r}+\theta p_{e}+\eta \tau \right). \end{array}$$

#### 2.2.3. Centralized Decision Model

The centralized decision model regards the leaguers in the supply chain structure as a whole, puts their interests in the second place, and maximizes the benefits in the whole supply chain as much as possible. According to this model, the optimal pricing decision can be specified [21–24].

**Proposition 1 .**

When $\eta <\sqrt{\rho \left(1-\theta \right)}$, *π*_Σ_^*c*^ is a concave function related to *p*_*e*_, *p*_*r*_, and *τ*. In the case that both retailers and suppliers are risk-neutral individuals, the optimal greenness of the product is shown in the following equation:

(7) $$\begin{array}{c} \tau^{c}=\frac{a\eta -2c\eta \left(1-\theta \right)}{2M}. \end{array}$$

The online and offline sales prices of the product are as follows:

(8) $$\begin{array}{c} p_{e}^{c}=\frac{1-s+\theta s}{2\left(1-\theta^{2}\right)}a+\frac{a\eta^{2}-2c\eta^{2}\left(1-\theta \right)}{4\left(1-\theta \right)M}+\frac{c}{2},\\ p_{r}^{c}=\frac{s+\theta -\theta s}{2\left(1-\theta^{2}\right)}a+\frac{a\eta^{2}-2c\eta^{2}\left(1-\theta \right)}{4\left(1-\theta \right)M}+\frac{c}{2}. \end{array}$$

where *M*=*ρ*(1 − *θ*) − *η*^2^. The proof process is as follows.

The centralized decision model seeks to maximize the benefit of the whole supply chain, so this decision model will be affected by the online product sales price *p*_*e*_^*c*^, offline product sales price *p*_*r*_^*c*^, the product greenness *τ*^*c*^, and other factors. According to the above hypotheses, the overall profit utility in the supply chain structure can be expressed as follows:

(9) $$\begin{array}{c} U^{c}\left(\Pi_{z}\right)=\left(p_{r}-c\right)\left(sa-p_{r}+\theta p_{e}+\eta \tau \right)+\left(p_{e}-c\right)\left[\left(1-s\right)a-p_{e}+\theta p_{r}+\eta \tau \right]-\frac{1}{2}p\tau^{2}. \end{array}$$

Since the centralized decision model regards the members in the supply chain structure as a whole, the wholesale price, as an internal variable, does not affect the overall income. Therefore, equation (9) does not include the wholesale price. The first derivatives of equation (9) about *τ*, *p*_*e*_, and *p*_*r*_ are as follows:

(10) $$\begin{array}{c} \frac{\partial U^{c}\left(\Pi_{z}\right)}{\partial \tau }=\eta \left(p_{r}-c\right)+\eta \left(p_{e}-c\right)-\rho \tau =\eta \left(p_{r}+p_{e}-2c\right)-\rho \tau ,\\ \frac{\partial U^{c}\left(\Pi_{Z}\right)}{\partial p_{e}}=\left(1-s\right)a+2\theta p_{r}-2p_{e}+\eta \tau +\left(1-\theta \right)c,\\ \frac{\partial U^{c}\left(\Pi_{z}\right)}{\partial p_{r}}=sa-2p_{r}+2\theta p_{e}+\eta \tau +\left(1-\theta \right)c. \end{array}$$

Accordingly, the Hessian matrix of the overall profit of the supply chain structure about *τ*, *p*_*e*_, and *p*_*r*_ can be written as follows:

(11) $$\begin{array}{c} H=\left(\begin{array}{ccc} -2 & 2\theta & \eta \\ 2\theta & -2 & \eta \\ \eta & \eta & -\rho \end{array}\right). \end{array}$$

If |*H*| < 0, then there is $\eta <\sqrt{\rho \left(1-\theta \right)}$. If *∂U*^*c*^(*II*_*Z*_)/*∂τ*=0, *∂U*^*c*^(Π_*Z*_)/*∂w*=0, and *∂U*^*c*^(Π_*z*_)/*∂p*_*e*_=0, then the optimal greenness of the product and the online and offline sales price can be obtained when the overall revenue of the supply chain is maximum.

**Corollary 1 .**

In this model structure, the demand of retail channels does not affect the greenness of products, but it is inversely proportional to the sales price of online products and positively proportional to the sales price of offline products [25]. The proof process is as follows:

The first-order derivative of the ratio of the offline sales channel demand *s* to the online sales price *p*_*e*_^*c*^ is obtained, as shown in the following equation:

(12) $$\begin{array}{c} \frac{\partial p_{e}^{c}}{\partial s}=\frac{\theta -1}{2\left(1-\theta^{2}\right)}a. \end{array}$$

Because 0 < *θ* < 1, *∂p*_*e*_^*c*^/*∂s* < 0.

The first-order derivative of the ratio of the offline sales channel demand *s* to the offline sales price *p*_*r*_^*c*^ can be presented as follows:

(13) $$\begin{array}{c} \frac{\partial p_{r}^{c}}{\partial s}=\frac{1-\theta }{2\left(1-\theta^{2}\right)}. \end{array}$$

Since 0 < *θ* < 1, *∂p*_*r*_^*c*^/*∂s* > 0.

Corollary 1 shows that since the centralized decision model considers the alliance members in the supply chain structure as a whole, the decision-making is analyzed from the perspective of the whole. Meanwhile, the offline market share as an endogenous variable does not affect the greenness of the product. When the offline market accounts for a relatively large proportion of consumers, the purchase channel of consumers is mainly physical retail stores. In this case, retailers may improve customer satisfaction through after sales and other means, but the offline market accounting for a large proportion of consumers may cause the phenomenon of short supply, thus raising the sales price of offline products.

### 2.3. Two-Channel Supply Chain Model for Fresh Agricultural Products

The development of society is inevitably accompanied by the improvement of people's material conditions and consumption levels, which prompts the masses to have an increasingly intense demand for fresh food and stricter quality pursuits. The development of “Internet + agriculture” and cold chain logistics technology makes the sales methods and sales environment of fresh agricultural products no longer simply rely on traditional offline channels. To improve corporate profits, reduce losses, and diversify consumers' purchasing forms, enterprises choosing to adopt the coexistence of online and offline channels to sell fresh agricultural products have sprung up. For example, fresh agricultural product suppliers (farmers, cooperatives, production bases, etc.) sell products through traditional retail channels on the one hand, and open online direct sales stores on Taobao, JD.com, Yihaodian, and other e-commerce platforms on the other hand to sell products. However, the addition of online channels will definitely impact the traditional sales form and transaction environment, which will undoubtedly exacerbate channel conflicts and the double marginal effect of supply chain members blindly seeking the best goals for themselves. Therefore, further research is needed on whether the introduction of direct online sales channels affects the state of supply chain coordination. However, in the current study, a way needs to be found that can effectively facilitate, coordinate, and improve the expected benefits of the supply chain.

The freshness of fresh agricultural products directly reflects the quality of the products, and the cross price between the selling price and the channel will also directly determine the occurrence of consumers' purchasing behavior. Therefore, to reflect consumers' demand for fresh agricultural products, the influence of these factors must be considered together. Among them, the distribution model of fresh produce A-type online and offline channel supply chain means that the supplier will wholesale fresh produce offline to retailers while also opening an online direct sales channel to sell some products directly to consumers. After analyzing the established model using the inverse method, the revenue sharing contract strategy is considered to be used to coordinate the management of the supply chain. After obtaining the range of contract parameters and proving that referring to the contract parameters can make the profits of each member and the whole of the supply chain better than the profits without contract constraints. It can be concluded that the use of revenue sharing contract strategy can promote the best supply chain benefits and improve the effectiveness of supply chain collaboration.

#### 2.3.1. Model Assumptions and Parameter Definitions

The present work studies a two-stage supply chain of fresh agricultural products with two channels, in which the supplier has the first-mover advantage. For the convenience of analysis, the following hypotheses are proposed in this study.

  Hypothesis 1: retailers order fresh produce from suppliers near the peak selling season. Consumers purchase products in only one channel during a sales cycle.
  Hypothesis 2: here, only the production cost of the supplier is considered, other costs are temporarily excluded, and it is assumed that the product has no residual value [26].
  Hypothesis 3: under rational and risky circumstances, retailers and suppliers make decisions to maximize their interests.
  Hypothesis 4: the potential demand of the market is not affected by online channels, and sellers can choose the channels of product purchase at will [27].

For the convenience of analysis, variable symbols used in this section are summarized: *ω* refers to the wholesale price determined by suppliers; *p*_1_ and *p*_3_ represent offline and online sales prices of retailers; *p*_2_ denotes supplier's online sales price; *θ*_0_ signifies the initial freshness of the product; *ε* stands for supplier's level of effort to maintain product freshness; *η* denotes the sensitivity coefficient of product freshness to time; *T* represents the sales cycle; *θ* indicates the market share of online sales channels; *k* describes the sensitivity coefficient of product preservation cost to preservation effort level; *α* denotes the cross-price sensitivity coefficient of online and offline channels and 0 < *α* < 1. Besides, *β* denotes the sensitivity coefficient of product freshness and 0 < *β* < 1; *a* represents the market size; *c*_0_ signifies the production cost of each unit of product produced by the supplier; *q*_1_ and *q*_3_ represent sales volume of retailers' offline and online channels, respectively; *q*_2_ denotes sales volume of suppliers' online channels; *π*_*m*_ and *π*_*r*_ represent profits of suppliers and retailers; *π*_*c*_ denote the total profit of the supply chain when centralized decisions are made.

#### 2.3.2. Model Construction and Solution Process

In the process of constructing the consumer demand function, it is necessary to consider the influence of two factors, namely, the degree to which consumers' purchase intention is affected by the freshness of fresh agricultural products and the degree to which market demand is affected by the price [28, 29]. Here, the demand of consumers is described through the classical linear demand, and the demand function of online and offline channels is expressed as follows:

(14) $$\begin{array}{c} d_{1}\left(p,t\right)=\theta a-p_{1}+\alpha p_{2}+\beta \theta \left(t\right), \end{array}$$

(15) $$\begin{array}{c} d_{2}\left(p,t\right)=\left(1-\theta \right)a-p_{2}+\alpha p_{1}+\beta \theta \left(t\right). \end{array}$$

When the utility of the product is not less than 0, consumers will buy the product. Therefore, the product sales volume of retailers' offline sales channel and suppliers' online sales channel at a certain time can be expressed as follows:

(16) $$\begin{array}{c} q_{1}=\int_{0}^{T}\left[\theta a-p_{1}+\alpha p_{2}+\beta \theta \left(t\right)\right]\text{d}t=\int_{0}^{T}\left[\theta a-p_{1}+\alpha p_{2}+\beta \left(\theta_{0}e-\eta t\right)\right]\text{d}t,\\ q_{2}=\int_{0}^{T}\left[\left(1-\theta \right)a-p_{2}+\alpha p_{1}+\beta \theta \left(t\right)\right]\text{d}t=\int_{0}^{T}\left[\left(1-\theta \right)a-p_{2}+\alpha p_{1}+\beta \left(\theta_{0}e-\eta t\right)\right]\text{d}t. \end{array}$$

Based on the above assumptions, profits of suppliers and retailers can be written as follows:

(17) $$\begin{array}{c} \pi_{m}=\left(p_{2}-c_{0}\right)q_{2}+\left(\omega -c_{0}\right)q_{1}-\frac{ke^{2}}{2},\\ \pi_{r}=\left(p_{1}-\omega \right)q_{1}. \end{array}$$

Assuming that retailers and suppliers in the dual channels of agricultural products cooperate to maximize the profits of the whole supply chain structure, the total profits of the supply chain system can be expressed as follows:

(18) $$\begin{array}{c} \pi_{c}=\left(p_{2}-c_{0}\right)q_{2}+\left(p_{1}-c_{0}\right)q_{1}-\frac{ke^{2}}{2}\\ =\left(p_{2}-c_{0}\right)\int_{0}^{T}\left[\left(1-\theta \right)a-p_{2}+\alpha p_{1}+\beta \left(\theta_{0}e-\eta t\right)\right]\text{d}t\\ +\left(p_{1}-c_{0}\right)\int_{0}^{T}\left[\theta a-p_{1}+\alpha p_{2}+\beta \left(\theta_{0}e-\eta t\right)\right]dt-\frac{ke^{2}}{2}. \end{array}$$

In this decision-making form, the Hessian matrix of the total profit of the supply chain regarding the online and offline sales price of the supply chain is shown in the following equation:

(19) $$\begin{array}{c} H_{2}=\left(\begin{array}{cc} \frac{\partial^{2}\pi_{c}}{\partial p_{2}^{2}} & \frac{\partial^{2}\pi_{c}}{\partial p_{2}p_{1}}\\ \frac{\partial^{2}\pi_{c}}{\partial p_{1}p_{2}} & \frac{\partial^{2}\pi_{c}}{\partial p_{1}^{2}} \end{array}\right)=\left(\begin{array}{cc} -2T & 2T\alpha \\ 2T\alpha & -2T \end{array}\right). \end{array}$$

According to the joint solution and simplification through *∂π*_*c*_/*∂p*_1_=0 and *∂π*_*c*_/*∂p*_2_=0, the optimal price of offline and online sales channels of the supply chain under centralized decision is finally obtained, as shown in the following equations:

(20) $$\begin{array}{c} p_{1}^{c*}=\frac{c_{0}}{2}+\frac{\beta \left(\left(\theta_{0}e-\eta T\right)/2\right)}{2\left(1-\alpha \right)}+\frac{\alpha a+\theta a-\alpha \theta a}{2\left(1-\alpha^{2}\right)}, \end{array}$$

(21) $$\begin{array}{c} p_{2}^{c*}=\frac{c_{0}}{2}+\frac{\beta \left(\left(\theta_{0}e-\eta T\right)/2\right)}{2\left(1-\alpha \right)}+\frac{a-\theta a+\alpha \theta a}{2\left(1-\alpha^{2}\right)}. \end{array}$$

Substituting equations (20) and (21) into equation (18), the maximum profit of supply chain system under the centralized decision model can be determined as follows:

(22) $$\begin{array}{c} \pi_{c}^{*}=T\frac{\beta \left(\theta_{0}e-\left(\eta T/2\right)\right)\left(a+\beta \left(\theta_{0}e-\left(\eta T/2\right)\right)\right)}{2\left(1-\alpha \right)}-c_{0}\beta \left(\theta_{0}e-\frac{\eta T}{2}\right)\\ +\frac{2\alpha \theta a^{2}\left(1-\theta \right)+a^{2}\left(\theta^{2}+{\left(1-\theta \right)}^{2}\right)}{4\left(1-\alpha^{2}\right)}+\frac{c_{0}^{2}\left(1-\alpha \right)-c_{0}a}{2}. \end{array}$$

#### 2.3.3. Supply Chain Coordination Mechanism under the Price Discount Contract

In the supply chain model of retailer opening online channels discussed in this study, suppliers assume the main coordinating responsibility, and the price discount contract sets the wholesale price determined by the supplier, which is related to the supplier's online sales channel, as shown in the following equation:

(23) $$\begin{array}{c} \omega \left(p_{2}\right)=c_{0}+\lambda \left(p_{2}-c_{0}\right). \end{array}$$

In equation (23), *λ* denotes the price discount coefficient and 0 < *λ* < 1.

When the supplier raises products' online sales price, the online sales channel will decline, and the wholesale price set by suppliers will rise. To ensure their profits, retailers will correspondingly raise the sales price of products in online and offline channels, which will enhance consumers' desire to buy in the online sales channels provided by suppliers. On the contrary, when the supplier reduces the online sales price of the product, the sales volume of the supplier's online sales channel will be increased, and the wholesale price determined by the supplier will be reduced. To attract consumers, the retailer will also reduce the online and offline sales price of the product [5, 30, 31]. Therefore, the price discount contract will not cause the situation that there is only single-channel demand in the supply chain system.

Profits earned by suppliers and retailers under this contract model can be expressed as follows:

(24) $$\begin{array}{c} \pi_{m}^{p}=\left(p_{2}-c_{0}\right)q_{2}+\left[\omega \left(p_{2}\right)-c_{0}\right]\left(q_{1}+q_{3}\right)-\frac{ke^{2}}{2},\\ \pi_{r}^{p}=\left[p_{1}-\omega \left(p_{2}\right)\right]q_{1}+\left[p_{3}-\omega \left(p_{2}\right)\right]q_{3}. \end{array}$$

### 2.4. Case Study on Double-Channel Supply Chain Coordination

Because the model structure is too complex, this study verifies the correctness of the model through specific example analysis to have a clearer understanding of the relationship between the supply chain and price discount strategy. By referring to a large number of literature, the values of each parameter are finally determined as follows: *α*=100, *θ*=0. 6, *c*_0_=10, *T*=10, *β*=0. 4, *η*=0. 5, *θ*_0_=0. 8, *k*=100, and *e*=5.

### 2.5. Analysis of the Influence of the Discount Coefficient on Supply Chain

#### 2.5.1. Influence of Discount Coefficient on Supply Chain Profit When Ignoring Compensation Cost

Price discount coefficients have a certain impact on supplier's profit and retailer's profit.  Figure 4 shows the analysis results of the total profit and profit of each member in the supply chain system at different price discount rates.

According to Figure 4, under the influence of price discount contracts, retailers' profits have increased and suppliers' profits have decreased to some extent, but the total profits have not been affected. After coordination, the total profits still keep a steady trend of rising. Besides, in the case of increasing price discount coefficient, compared with retailers, suppliers' profits change significantly more. Because *λ*=*α*/(1 − *α*), when the price discount coefficient increases, the dual-channel price crossover coefficient is proportional to the profits of suppliers and retailers without contract coordination. In other words, when the dual-channel price crossover coefficient keeps rising, the profits of suppliers and retailers also keep rising.

In a word, retailer revenue and total system revenue increase obviously with the increase in price discount coefficient after the price discount strategy is applied. Therefore, the coordination effect of the price discount contract is more obvious compared with that of the contract constraint, and the profits obtained by members in the supply chain system continue to rise with the growth of the price discount coefficient. However, it should be noted that after the introduction of a price contract mechanism, the profits of some members in the supply chain system may not rise. Therefore, to increase the profits of all members, further profit distribution is required.

#### 2.5.2. Influence of Discount Coefficient on Supply Chain Profit When Compensation Cost Is Fixed

To improve the acceptance of each member of the supply chain system to the price discount contract, after the profit increases, the retailer will provide the supplier with additional compensation expense P, and the compensation expense is fixed at 4,500. In this case, the profit of the retailer and the supplier is $\hat{\Delta \pi_{m}^{p*}}=\pi_{m}^{p*}+P$ and $\hat{\Delta \pi_{r}^{p*}}=\pi_{r}^{p*}+P$, respectively, as shown in Figure 5.

From Figure 5, when the compensation cost is kept at a certain value, the increase in price discount coefficient makes the growth of retailer's profit continuously increase, while the increase in supplier's profit keeps decreasing. Therefore, when the compensation cost is fixed, the increase in price discount coefficient has a favorable effect on retailers, but the interests of suppliers are damaged to a certain extent.

#### 2.5.3. Impact of Compensation Costs on Supply Chain Profits

The price discount rate is assumed to be a certain value of 0.5 to explore the variation trend of supply chain profit with compensation cost, and the results are shown in Figure 6.

From Figure 6, when the price discount coefficient is fixed, the increase in compensation cost leads to a gradual increase in the profit gap of suppliers before and after contract coordination. However, the profit gap of retailers before and after contract coordination keeps decreasing, and the total profit gap of the whole supply chain system remains unchanged. The main cause of this phenomenon is that the main purpose of the increase of compensation cost is to reallocate the profits of all members of the supply chain after the price discount contract is used; since the total profit of the supply chain system is consistent with the total profit of the supply chain system under centralized decision-making, it will not change, but the profit of suppliers and retailers will be affected by compensation costs to a certain extent.

When the compensation cost is between 1,000 and 3,000, the profit of retailers in the supply chain system will be improved by using the price coordination mechanism, while the profit of suppliers will be reduced to some extent. When the value of compensation cost is 7,000–9,000, applying the price coordination mechanism will increase the profit of suppliers in the supply chain system, while the profit of retailers will decline to a certain extent. This is because the above condition does not satisfy the constraint of *Pϵ*(*T*[*a* − 2*c*_0_ − *sa*+4*c*_0_*α*+*β*(*θ*_0_*e* − *ηT*/2)]^2^/16(1 − *α*), 3*T*[*a* − 2*c*_0_ − *sa*+4*c*_0_*α*+*β*(*θ*_0_*e* − *ηT*/2)]^2^/32(1 − *α*)). When the compensation cost is between 4,000 and 6,000, the profit of both retailers and suppliers will increase. Therefore, a reasonable design of compensation cost can effectively improve the profit of retailers and suppliers, thus maximizing the profit of the whole supply chain system.

### 2.6. Analysis of the Effect of Freshness on the Supply Chain

In this test, the price discount rate is fixed at 0.5, and the compensation cost is fixed at 4,500. The effect of freshness on the profit of each member in the supply chain system is investigated, and the results are shown in Figure 7.

From Figure 7, the improvement of the freshness of fresh agricultural products has a positive effect on the profit of retailers and meanwhile a negative effect on the total profit of suppliers and supply chain system. The reason for this phenomenon is that suppliers' efforts to keep their products fresh lead to excessive costs and reduced profits; however, the improvement in the product freshness increases product sales, so that retailers can obtain more profits. Therefore, to ensure the total profit, the insurance effort level needs to be controlled within a certain range.

The natural perishability of fresh agricultural products makes them prone to loss during production, transportation, and sale in the market. The improvement of people's material living conditions has made consumers more and more strict with the quality and safety requirements of fresh agricultural products. The method of selling products through the supply chain of online and offline channels effectively solves the problems of small influence of offline traditional circulation mode, asymmetric information, and many circulation links, and a reasonable supply chain coordination contract can promote the benefits of supply chain members to be as optimal as possible. The influence of information asymmetry in the direct sales of fresh agricultural products under the e-commerce environment is studied. Qiu et al. (2020) [32] proposed a three-level fresh agricultural product supply chain consisting of fresh agricultural product suppliers, logistics service providers, and large e-commerce platforms. Considering the perishability of fresh agricultural products, the impact of logistics space-time cost and freshness of fresh agricultural products on the profits of various stakeholders in the supply chain is analyzed. Three cases are considered: (1) complete information, (2) partial information, and (3) logistics space-time cost. Based on principal-agent theory and supply chain coordination contract theory, an analytical model is established to describe the impact of revenue sharing contract on the operation of fresh agricultural product supply chain. The modeling results denote that under the condition of complete information, the increase of the loss rate of fresh agricultural products is related to the decrease of the profit of fresh agricultural products supply chain.

## 3. Conclusions

In the face of increasingly severe environmental problems and the requirements of the government and consumers, enterprises are paying more and more attention to the green production and management of products. The development of e-commerce has broken through the traditional sales model of enterprises; that is, suppliers will not only sell products through offline retail channels, but also sell products through online direct sales channels.

The dual-channel supply chain has brought great convenience to consumers, but the opening of online transaction channel will inevitably bring some impact on the traditional sales model. Based on blockchain technology, the present work conducts coordinated management of the dual-channel supply chain. Then, under the background that both retailers and suppliers are risk-neutral individuals, the benchmark model of dual-channel supply chain is constructed, and the online and offline sales prices of products under different decision-making modes are analyzed. Finally, taking fresh agricultural products as an example, the online and offline sales channels of fresh agricultural products are studied, and a dual-channel supply chain model is constructed. The profit and equilibrium price of each member in the supply chain system under this model is obtained by the inverse method. The research results manifest that when the compensation fee is fixed at 4500, the result of the increase of the price discount coefficient is that the profit increase of the supplier is gradually decreasing, while the profit increase of the retailer is increasing gradually. The other parameters remain unchanged, so that the price discount rate is 0.5. When the compensation fee increases from 1000 to 9000, the profit after the supplier coordination increases from 13175 to 21175, but the overall profit after coordination remains at 20150.

However, the dual-channel supply chain studied here is formed by a single retailer and supplier. In reality, the actual supply chain may be composed of multiple suppliers and retailers, or there are other channel members, which will become the focus of subsequent research.

## Figures and Tables

**Figure 1:** Blockchain infrastructure.

**Figure 2:** Structure of the data layer.

**Figure 3:** Decision-making process of supply chain leaguers.

**Figure 4:** Changes in profits when compensation costs are ignored. (a) The influence of discount coefficient on the profit of supply chain system; (b) profit changes before and after the coordination.

**Figure 5:** Profit changes when compensation costs are fixed. (a) The influence of discount coefficient on the profit of supply chain system; (b) profit changes before and after coordination.

**Figure 6:** Variation trend of supply chain profit with compensation cost. (a) The impact of compensation costs on the profit of the supply chain system; (b) profit changes before and after coordination.

**Figure 7:** Variation trend of supply chain profit with the product freshness. (a) The impact of the product freshness on the profit of the supply chain system; (b) profit changes before and after coordination.

## Data Availability

The data used to support the findings of this study are included within the article.

## References

[1] Zhu Z., Bai Y., Dai W., Liu D., Hu Y. (2021). Quality of e-commerce agricultural products and the safety of the ecological environment of the origin based on 5G Internet of Things technology. *Environmental Technology & Innovation*.

[2] Singh A., Mankotia D. S., Irshad M. (2017). A single-step multiplex quantitative real time polymerase chain reaction assay for hepatitis C virus genotypes. *Journal of translational internal medicine*.

[3] Mu Z., Liu X., Li K. (2020). Optimizing operating parameters of a dual E-commerce-retail sales channel in a closed-loop supply chain. *IEEE Access*.

[4] Singh A., Jenamani M., Thakkar J. J., Rana N. P. (2021). Propagation of online consumer perceived negativity: quantifying the effect of supply chain underperformance on passenger car sales. *Journal of Business Research*.

[5] Qi Q., Wang J., Xu J. (2018). A dual-channel supply chain coordination under carbon cap-and-trade regulation. *International Journal of Environmental Research and Public Health*.

[6] Zhang X.-M., Li Y.-Y., Liu Z., Li Q.-W., Wang J. (2021). Coordination contracts of dual-channel supply chain considering advertising cooperation. *International Journal of Information Systems and Supply Chain Management*.

[7] Miraz M. H., Ali M. (2018). Applications of blockchain technology beyond cryptocurrency. *Annals of Emerging Technologies in Computing*.

[8] Chen G., Xu B., Lu M., Chen N.-S. (2018). Exploring blockchain technology and its potential applications for education. *Smart Learning Environments*.

[9] Sikorski J. J., Haughton J., Kraft M. (2017). Blockchain technology in the chemical industry: machine-to-machine electricity market. *Applied Energy*.

[10] Zhang Y., Wen J. (2017). The IoT electric business model: using blockchain technology for the internet of things. *Peer-to-Peer Networking and Applications*.

[11] Angraal S., Krumholz H. M., Schulz W. L. (2017). Blockchain technology. *Circulation: Cardiovascular Quality and Outcomes*.

[12] Ichikawa D., Kashiyama M., Ueno T. (2017). Tamper-resistant mobile health using blockchain technology. *JMIR mHealth and uHealth*.

[13] Benchoufi M., Ravaud P. (2017). Blockchain technology for improving clinical research quality. *Trials*.

[14] Biktimirov M. R., Domashev A. V., Cherkashin P. A., Shcherbakov A. Y. (2017). Blockchain technology: universal structure and requirements. *Automatic Documentation and Mathematical Linguistics*.

[15] Gaggioli A. (2018). Blockchain technology: living in a decentralized everything. *Cyberpsychology, Behavior, and Social Networking*.

[16] Li G., Zheng H., Liu M. (2019). Reselling or drop shipping: strategic analysis of E-commerce dual-channel structures. *Electronic Commerce Research*.

[17] Wiseman A. E., Ellig J. (2017). Market and nonmarket barriers to internet wine sales: the case of Virginia. *Business and Politics*.

[18] Chen M.-S., Lan C.-H. (2001). Dynamic production plan of probabilistic market demand and fixed selling time with unreliable machines and obtainable working hour capacity. *Journal of the Operations Research Society of Japan*.

[19] Anning-Dorson T. (2017). Moderation-mediation effect of market demand and organization culture on innovation and performance relationship. *Marketing Intelligence & Planning*.

[20] Ulusoy V., Demiralay S. (2017). Energy demand and stock market development in OECD countries: a panel data analysis. *Renewable and Sustainable Energy Reviews*.

[21] Lintner P. (2017). De/centralized decision making under the European resolution framework: does meroni hamper the creation of a European resolution authority?. *European Business Organization Law Review*.

[22] Charalambous C. D., Ahmed N. U. (2017). Centralized versus decentralized optimization of distributed stochastic differential decision systems with different information structures-Part I: a general theory. *IEEE Transactions on Automatic Control*.

[23] Liu Z., Lang L., Hu B., Shi L., Huang B., Zhao Y. (2021). Emission reduction decision of agricultural supply chain considering carbon tax and investment cooperation. *Journal of Cleaner Production*.

[24] Li H., Wang C., Shang M., Ou W. (2017). Pricing, carbon emission reduction, low-carbon promotion and returning decision in a closed-loop supply chain under vertical and horizontal cooperation. *International Journal of Environmental Research and Public Health*.

[25] Xiang B., Elias J., Martignon F., Di Nitto E. (2021). Resource calendaring for mobile edge computing: centralized and decentralized optimization approaches. *Computer Networks*.

[26] Andersen P. H., Drejer I., Østergaard C. R., Søberg P. V., Wæhrens B. V. (2019). Supplier value creation configurations in high-cost countries. *Journal of Global Operations and Strategic Sourcing*.

[27] Nagasawa K., Davidson F. T., Lloyd A. C., Webber M. E. (2019). Impacts of renewable hydrogen production from wind energy in electricity markets on potential hydrogen demand for light-duty vehicles. *Applied Energy*.

[28] Patra P. (2018). Distribution of profit in a smart phone supply chain under Green sensitive consumer demand. *Journal of Cleaner Production*.

[29] Amir R., Erickson P., Jin J. (2017). On the microeconomic foundations of linear demand for differentiated products. *Journal of Economic Theory*.

[30] Xu J., Qi Q., Bai Q. (2018). Coordinating a dual-channel supply chain with price discount contracts under carbon emission capacity regulation. *Applied Mathematical Modelling*.

[31] Yang S., Liu H., Wang G., Hao Y. (2021). Supplier’s cooperation strategy with two competing manufacturers under wholesale price discount contract considering technology investment. *Soft Computing*.

[32] Qiu F., Hu Q., Xu B. (2020). Fresh agricultural products supply chain coordination and volume loss reduction based on strategic consumer. *International Journal of Environmental Research and Public Health*.

